# Transcultural validation of the “revised sport motivation scale” (SMS‐II) in Arabic language: Exploratory study on motivation in sport for a sample of Tunisian Athletes

This article has been retracted.

**DOI:** 10.1371/journal.pone.0295262

**Published:** 2023-11-30

**Authors:** Mohamed Baaziz, Ali Aloui, Amel Tayech, Matthew Stults-Kolehmainen, Mohamed Arbi Mejri, Abderraouf Ben Abderrahman

**Affiliations:** 1 Higher Institute of Sport and Physical Education of Ksar-Said, University of Manouba, Manouba, Tunisia; 2 Higher Institute of Sport and Physical Education of Gafsa, University of Gafsa, Gafsa, Tunisia; 3 Tunisian Research Laboratory “Sports Performance Optimization”, National Center of Medicine and Science in Sports (CNMSS), Tunis, Tunisia; 4 Division of Digestive Health, Yale New Haven Hospital, New Haven, CT, United States of America; 5 Department of Biobehavioral Sciences, Teachers College-Columbia University, New York, NY, United States of America; National Cheng Kung University College of Medicine, TAIWAN

## Abstract

**Background:**

Sports performance is the result of an interaction of several variables, such as physical, technical, and psychological. The ability of athletes to use motivation, is an important predictor to achieve high performance in sport. SMS‐II comprised 18 elements to measure six behavioral control factors.

**Aim:**

This study aims to validate an Arabic version of the revised sports motivation scale‐II (SMS‐II) and measure the psychometric properties of factorial structure, internal reliability, construct validity, and sensitivity.

**Methods:**

A total of 780 athletes from different disciplines (432 men, 348 women; mean age = 18.97 years) participated in this study. Athletes voluntarily responded to the version of SMS‐II. Factorial validity was established by principal component analysis. Both exploratory (EFA; *N* = 390; males: 52.6%; females: 47.4%; [13–18] = 172; [19–30] = 218) and confirmatory (CFA; *N* = 390; males: 58.2%; females: 41.8%; [13–18] = 247; [19–30] = 143) analyses were examined.

**Results:**

The 18 SMS-II items revealed perfect reliability (McDonald’s omega = 0.841, Cronbach’s α = 0.858, Gutmann’s λ6 = 0.952) and good temporal stability (ICC = 0.960, 95% CI = 0.915–0.980; *r* = 0.935, 95% CI = 0.889–0.963 at *p* < 0.001) over 4-week period. The CFA adjustment indices were perfect.

**Conclusion:**

The results tended to clarify all indices as perfect adjustments to the theoretical model, ensuring the confirmation of factor structure and construction validity regarding the Tunisian sports workforce.

## Introduction

Self Determination Theory (SDT) is a theory of human motivation that concerns people’s inherent growth tendencies and psychological need. SDT has been extensively used in sports. Some concepts examined using this theory includes: coaching styles, the psychological needs of athletes, and the principles of motivation. Coaches’ behaviors lead to athletes’ motivation and their subsequent needs by influencing levels of commitment, psychological well-being, and athletic performance [1]. Therefore, the variables of motivation and sports activities change according to the context. This implies that the frequency of these activities will be higher when athletes engage in situations that are better suited to their motivations and objectives [2]. The SDT presents a continuum from self-determination through controlled motivation to self-motivation. Intrinsic motivation has an important place in the field of human motivation [3–8]. Deci and Ryan confirm that intrinsic motivation increases by internal, autonomous regulation without external intervention. Hence, intrinsically motivated people also feel self-determined and extrinsic motivation comes from external regulation controlled [9,10].

In the same sense, the SDT identifies four forms of extrinsic motivation regulation: external control (i.e., behavior controlled by external factors); introjected regulation (i.e., the activity depends on the obligation of an individual or a group to continue); identified regulation (i.e., close to self-determination, due to positive repercussions); and integrated regulation (i.e., the most self-determined, sport is important to the athlete) [11]. Amotivation does not bring any conformity with self-determination [12]. It is presented as a total absence of integrated regulation. It should be noted that extrinsic and intrinsic motivations are the main axes of self-determination theory [9,10,13].

In fact, SDT varies depending on the degree of internalization in relation to different types of behavioral integration (i.e., external regulation, introjected regulation, identified regulation, and integrated regulation) [14]. Several works [15,16] emphasize that this is a theoretical framework allowing the understanding of motivation according to several forms of behavioral regulation [9,17,18]. This theoretical model analyzes its different forms without the complexity of the concept of motivation by Vallerand and Grouzet [19]. Many studies have justified the three forms of motivation [11]. According to the continuum of self-determination, intrinsic motivation is the most self-determined form of motivation, whereas extrinsic motivation is indicated as the least self-determined type. Indeed, this continuum changes with the regulation of motivation (i.e., intrinsic, identified, introjected, external, and amotivation) [9,13].

There is a continuum, with different levels presenting different types of motivation. Brière, Vallerand [15] developed the Sport Motivation Scale (SMS-28) to measure the levels in sports as well as motivation based on the SDT. Pelletier, Tuson [11] validated the English version. The exploratory factor analysis (EFA) of the two instruments revealed seven factors: MI to knowledge, MI to stimulation, MI to fulfillment, external regulation, interjected regulation, identified regulation, and motivation. This scale has been translated into several languages. Both versions of the SMS did not include the integrated control measure [20] and therefore measures were taken to address the limitations of this instrument. Pelletier, Vallerand [21] have developed SMS-6 by integrating a new measurement factor (i.e., integrated regulation). However, the results of the new element and the internal consistency of the sub-scales were inadequate to ensure the SMS-6 version. Pelletier, Rocchi [20] (Sports Motivation Scale-II) and Pelletier, Vallerand [21] (Global motivation scale) confirmed some limitations. Pelletier, Vallerand [21] proposed to include integrated regulation. These researchers suggested that some items should be scaled up and that intrinsic sub-scales should be unified into a single factor. They also proposed a revised version of the SMS-6.

Another study showed that the Behavioral Regulation in Sport Questionnaire (BRSQ) is an alternative measure of sports motivation based on SDT. In summary, both versions BRSQ-6 and BRSQ-8 aim to evaluate the regulations (i.e., integrated, identified, interjected, and external), the three forms of intrinsic motivation: stimulation, knowledge, and fulfillment and amotivation [22]. The BRSQ-6 contains the same forms and values of the overall intrinsic motivation rather than the three intrinsic motivations.

Pelletier, Rocchi [20] suggested a new English version of Sport Motivation Scale-II (SMS-II) that evaluates different forms of behavior regulation in the sports context within the framework of self-determination theory [13]. Several researchers [16,23,24] treated various psychometric properties of the instrument and concluded that this version is more reliable than the original SMS-28. Extensive studies by Pelletier and his collaborators have measured the psychometric properties of SMS-II in Canadian athletes. CFAs reported the creation of an 18-element scale assessing six factors of three items at each sub-scale (i.e., intrinsic motivation, integrated regulation, identified regulation, introjected regulation, external regulation, and amotivation). The SMS-II model was compared to the original version. In summary, the results indicated that this was more appropriate than the original scale. Therefore, the psychometric properties of SMS-II have been validated in Brazil [23], in Español hablado in Mexico [25], in Spanish for adolescent athletes [24], in Spanish [26], in French [16] in Malay [27].

The study of motivation in sports is currently scared in Arabic-speaking countries. The research of types of motivation in the sport context could help researchers and coaches in Arab countries to identify effective interventions that could develop athletes’ performance and experience. We will try to better understand the aspects that determine his motivation (i.e., intrinsic motivation, integrated regulation, identified regulation, introjected regulation, external regulation, and amotivation) among the athlete. Therefore, the objective of our study was to trans-culturally adapt and assess the factor structure, internal consistency, construct validity, and sensitivity of the revised sports motivation scale-II (SMS-II). To test the reliability of the translated and adapted tool, we followed a sub-sample of the all population of athletes for four weeks.

## Methods and equipment

### Population

Our sample consists of 780 athletes (432 men = 55.4% and 348 women = 44.6%; mean age = 18.97 years, SD = 4.01; 13 to 30). The population as a whole participates in various disciplines: 392 athletes in team sports (soccer, handball, volleyball, and basketball) and 388 athletes in individual sports (kick boxing, English boxing, Taekwondo, athletics, gymnastics, and swimming). Data from 780 questionnaires of 800 responses were obtained for final analysis; 20 were removed for missing responses. The geographical distribution of the athletes was as follows: Tunis (20.3%), Sfax (19.1%), Kairouan (26.7%), Gafsa (20%) and Gabes (14%) (the north of Tunisia (Tunis), the center of Tunisia (Sfax and Kairouan), and the south of Tunisia (Gafsa and Gabes)).

### Measurement

Pelletier, Rocchi [20] improved the SMS by creating the revised Sports Motivation Scale-II (SMS-II) as an alternative measure. These authors indicated that the SMS-II develops the defaults of the SMS, and they result that the SMS-II develops and assesses good psychometric properties to measure the level of motivation for sport than the original scale (SMS-28) by adding the integrated regulation. The scale was designed to assess athletes’ level of motivation for sport as a function of SDT. The SMS-II has justified good reliability for its subscales. The SMS-II consists of 18 items that are divided in to 6 subscales (namely, intrinsic motivation, integrated motivation, identified regulation, introjected regulation, external regulation, and amotivation) with three items for each dimension within the self‐determination theory to justify the use of motivation. All items were examined using a 7-point Likert scale ranging from 1 (Not at all true) to 7 (Very true). The highest numerical level represents the highest level of satisfaction. In the study, we have chosen this scale to measure motivation in a sample of Tunisian athletes.

### Procedure

In translation and validation, researchers suggest various procedures for questionnaires [28,29]. We use the translation and back-translation procedure to obtain the translation of the Arabic version of the SMS-II validated in English by Pelletier, Rocchi, Vallerand, Deci and Ryan [20]. This trans-cultural validation respected the International Test Commission (ITC) guidelines [30,31]. The translation of this scale (SMS-II) was carried out by two translation teams characterized by their in-depth knowledge of the source and target languages. First, the first team, consisting of two bilingual translators, translated the original version into Arabic. This produced two Arabic versions of the tool that were combined into a common version after a meeting between the authors to get the differences between the two versions. Then, two experienced English speakers who know Arabic very well, did the translation in reverse without the presence of the English version, which resulted in a version equivalent to the original version. In conclusion, no changes were made to the Arabic version. Finally, the implemented version was compared to the original article.

The administration of the questionnaire was done in 26 October 2021 following the start of the sports season and the end of the health crisis of coronavirus, 800 questionnaires were distributed. We informed the club coordinators of the objectives of the work. The scales were distributed to the teams before the training session. The SMS-II was completed two hours before the start of the athletic competitions. The instructions for the tool were well explained to the athletes. The athletes indicated their age, gender, and sport discipline.

The present work was fully validated by the ethics committee of the National Center of Medicine and Sports Sciences of Tunisia (approval number LR09SEP01) before the beginning of the analyses. For the minor athletes, we took for their parents’ permission. Verbal informed consent was collected from each athlete before starting the work. The participation of the athletes was voluntary. The raw data obtained by the participants were analyzed to ensure maximum confidentiality. All authors had access to information that could identify individual participants during or after data collection.

### Statistical analysis

The data normality was demonstrated with Skewness (Sk) values between (−0.611 and −1.307) and Kurtosis (Kr) values located (−0.378 and 1.666) (**Table 2**). Asymmetric values between +2 and −2 are considered acceptable for normal distribution [32,33]. Therefore, we can deduce that the distribution is normal.

To examine the psychometric quality of the scale, the Cronbach’s α, McDonald’s ω, and Gutmann’s λ6 evaluated the internal consistency of the sub-scales and the overall score of the instrument. The temporal stability of SMS-II was measured using the test-retest consistency index (Intra-Class Correlation, Bivariate correlations). Predictive validity was examined by measuring the correlation matrix and the Pearson correlation coefficient.

To analyze the factor structure of the scale, an orthogonal Varimax type exploratory factor analysis (EFA) such as Kaiser’s [34] Varimax criterion with a principal-component analysis (PCA) was used on our scale from the 18 items of the tool [35]. Each item was retained if the loading was equal to or greater than 0.40 [36]. Sampling adequacy was calculated by the Kaiser-Meyer-Olkin (KMO) and the Bartlett sphericity test (Bartlett test) [37,38]. It is suggested that the KMO test value be greater than 0.6 and the Bartlett test be correlated with a significant *p*-value [39].

A confirmatory factor analysis (CFA) of the first order with maximum likelihood estimation was verified the factor structure in six dimensions of SMS-II factors. The analyses addressed several indices measuring the fit efficiency of the model tested. The following indices were used to determine the models’ fit to the data collected. To measurement the goodness of fit of the model, we used the Goodness of Fit Index (GFI) [40–42], as well as its adjusted index (AGFI), which should be equal to or greater than 0.90 [43]. We then looked at the root mean square error of approximation (RMSEA). It should be ≤0.05 for a good fit [44]. Furthermore, we applied the standardized root mean square residual (SRMR), which should be less to equal than 0.10 for an acceptable fit [45]. Moreover, the Comparative Fit Index (CFI) [46], the Not Normed Fit Index (NNFI), the Normed Fit Index (NFI), the Parsimony Comparative Fit Index (PCFI) and the Parsimony NFI (PNFI) have been verified [47]. The CFI, NFI, TLI, PCFI, and PNFI values should be ≥0.95, the NFI value should be ≥0.90 [41]. A significant χ^2^ value relative to the degrees of freedom confirms that the proposed model is not supported by the observed data. Whereas the adequacy of the model to the collected data depends on a non-significant χ^2^ value [48]. The ratio of chi-square to degree of freedom (χ^2^/df) was performed to compare the fit indices among models. If χ^2^/df < 3, it means that the model fit is acceptable [49]. However, chi-square (χ^2^) is related to on the sample population. Also, the more complex the model tested, the more sensitive the χ ^2^ becomes [50].

Further, a sensitivity analysis (analysis of variance, ANOVA) was performed to examine the impact of age, gender, and sport type on the scores of each dimension of the instrument.

EFA was checked on a random split-half sample, whereas CFA was per-formed on the other split-half sample. EFA was measured by the commercial software "Statistical Package for Social Sciences" SPSS (version 25, IBM, Armonk, NY, USA) and the software programs JASP (Version 0.16.4.0), but CFA was calculated with AMOS (version 25, IBM, Armonk, NY, USA).

## Results

### Instrument quality

The basic characteristics of the sample population are shown in **Table 1**.

**Table 1:** Basic characteristics of the sample population.

Variable		Effective			Pourcentage (%)
Age		[13–18]	Total (*N* = 780)	419	53.70
			EFA (*n* = 390)	172	44.10
			CFA (*n* = 390)	247	63.30
			Test-retest (*n* = 51)	28	54.80
		[19–30]	Total (*N* = 780)	361	46.30
			EFA (*n* = 390)	218	55.90
			CFA (*n* = 390)	143	36.70
			Test-retest (*n* = 51)	23	45.20
Gender		Male	Total (*N* = 780)	432	55.40
			EFA (*n* = 390)	205	52.60
			CFA (*n* = 390)	227	58.20
			Test-retest (*n* = 51)	35	68.60
		Female	Total (*N* = 780)	348	44.60
			EFA (*n* = 390)	185	47.40
			CFA (*n* = 390)	163	41.80
			Test-retest (*n* = 51)	16	31.40
Type of sport		Individual sport	Total (*N* = 780)	388	49.70
			EFA (*n* = 390)	192	49.20
			CFA (*n* = 390)	196	50.30
			Test-retest (*n* = 51)	27	52.90
		Team sport	Total (*N* = 780)	392	50.30
			EFA (*n* = 390)	198	50.80
			CFA (*n* = 390)	194	49.70
			Test-retest (*n* = 51)	24	47.10
Governorates	Total (*N* = 780)	Tunis		158	20.30
		Sfax		149	19.10
		Kairouan		208	26.70
		Gafsa		156	20
		Gabes		109	14

The averages, standard deviations, kurtosis, and skewness of the SMS‐II items are shown in **Table 2**. Data were normally parted in terms of skewness and kurtosis.

**Table 2:** Descriptive statistics and normality of the 18-Item SMS-II.

Item	M	SD	Sk	Kr
1	5.58	1.52	-1.222	0.972
2	5.49	1.51	-1.158	0.794
3	5.54	1.45	-1.122	0.750
4	5.67	1.43	-1.185	0.862
5	5.59	1.38	-1.158	1.014
6	5.67	1.42	-1.177	0.875
7	5.70	1.40	-1.307	1.666
8	5.49	1.32	-1.003	1.023
9	5.64	1.35	-1.163	1.337
10	4.98	1.76	-0.647	-0.575
11	5.06	1.65	-0.696	-0.389
12	5.03	1.74	-0.688	-0.539
13	5.63	1.44	-1.088	0.511
14	5.46	1.36	-1.048	0.655
15	5.46	1.39	-0.977	0.384
16	4.86	1.79	-0.726	-0.453
17	4.79	1.79	-0.768	-0.378
18	4.86	1.78	-0.611	-0.713

*Note*. M, Mean; SD, Standard deviation; Sk, Skewness; Kr, Kurtosis.

Similarly, the averages and standard deviations of the SMS‐II sub‐scales by sex and kind sport are presented in **Table 3**.

**Table 3:** Means and standard deviations of the SMS‐II sub-scales by sex and kind of sport (i.e., individual versus team sports).

Sex	Sport		IM	Int.M	Id.R	Intro.R	ER	AM
[13–18]	Individual sport	M	16.31	17.23	16.51	15.22	16.52	14.10
		SD	4.53	3.93	3.57	4.65	3.82	5.19
	Team sports	M	16.99	17.82	17.03	16.41	16.83	14.75
		SD	4.22	3.71	3.98	4.35	4.13	5.11
[19–30]	Individual sport	M	16.66	16.17	16.29	13.56	16.08	14.36
		SD	4.22	4.04	3.73	5.20	4.31	5.26
	Team sports	M	16.59	16.75	17.39	15.32	16.79	14.82
		SD	4.18	4.07	3.30	4.59	3.61	4.95

*Note*. M, Mean; SD, Standard deviation; IM, intrinsic motivation; Int.M, integrated regulation; Id.R, identified regulation; Intro.R, introjected regulation; ER, external regulation; AMO, amotivation.

The stability over time of the SMS-II was assessed using the test-retest consistency index. A sports group of 51 athletes (35 men, 16 women; mean age = 19.41 years, SD = 4.64) responded to the scale. 4-week later, these participants filled out the same scale. The test-retest sample is included in the overall study population. This was a homogeneous population in terms of age and gender. Furthermore, our results presented that the SMS-II [20] had good temporal stability (ICC = 0.960, 95% CI = 0.915–0.980; *r* = test and retest = 0.935, 95% CI = 0.889–0.963 at *p* < 0.001). The temporal stability (test-retest reliability) of the SMS-II was examined by correlational analysis between SMS-II scores obtained by 51 individuals on two occasions 4-week intervals. A minimum sample size of 22 subjects is required to detect an ICC value of 0.50 for 80% power with an alpha fixed at 0.05 [51]. In case of possible dropout in the retest phase, an additional twenty percent of the minimum sample is proposed, resulting in a target number of 27 subjects. Hence, the number of 51 athletes was sufficient to verify the tool’s temporal stability. Therefore, the intraclass coefficient (ICC) was 0.847, showing excellent temporal stability of the instrument. The correlation coefficient was .935 (*p* < 0.001), indicating perfect temporal stability of the scale. The test-retest reliability data determined by the correlations between the values of SMS-II as a function of time are presented in **Table 4**.

**Table 4:** The test-retest reliability of the sports motivation scale SMS-II (*n* = 51).

	Test-retest reliability	
	Intra-class correlation	Bivariate correlations
SMS-II (CI 95%)	0.960 (0.915–0.980)	0.935*** (0.889–0.963)

*Note*. *** Statistically significant at *p* < 0.001.

Composite scores of test-retests had varying degrees of association by both measurements, with the largest significant association being between Intro.R and MI (*r* = 0.37 at *p* < 0.01) See **Fig 1**. Most of the factors are associated with the dominant dimension IM, which justifies the adding the integrated subscale and the creation of one measure of intrinsic motivation. This result is consistent with result of Pelletier, Rocchi [20].

**Fig 1:** Pearson’s heatmap. Averaged across all motivational factors were positively correlated (0.32< *r* <0.37, *p* < 0.05) and only significant association being between amotivation and intrinsic motivation (*r* = -0.28, *p* < 0.05).

Predictive validity was evaluated by measuring the Pearson correlation. The results of the correlation matrix between the 18 statements of the SMS-II indicated a positive correlation at *p* < 0.001 between most variables. The coefficient *r* was between 0.101 and 0.873. For some items, correlations were good, for example the correlation between item 11 ("Because I feel better about myself when I do") and item 12 ("Because I would not feel worthwhile if I did not") (*r* = 0.873 at *p* < 0.001), as well as the correlation be-tween item 16 ("So that others will praise me for what I do") and item 17 ("It is not clear to me anymore; I don’t really think my place is in sport") (*r* = 0.873 at *p* < 0.001). However, some coefficients were small, such as the coefficient on the correlation between item 9 ("Because I found it is a good way to develop aspects of myself that I value") and item 18 ("I used to have good reasons for doing sports, but now I am asking myself if I should continue ") (*r* = 0.101 at *p* < 0.04), as well as the coefficient of the correlation between item 5 ("Because through sport, I am living in line with my deepest principles ") and item 9 ("Because I found it is a good way to develop aspects of myself that I value ") (*r* = 0.110 at *p* < 0.03) (**Table 5**).

**Table 5:** Correlations between the 18-Item SMS‐II.

		1	2	3	4	5	6	7	8	9	10	11	12	13	14	15	16	17	18
Item 1	*r*	1																	
	P																		
Item 2	*r*	0.871	1																
	P	<0.001																	
Item 3	*r*	0.836	0.868	1															
	P	<0.001	<0.001																
Item 4	*r*	0.240	0.263	0.272	1														
	P	<0.001	<0.001	<0.001															
Item 5	*r*	0.253	0.293	0.289	0.824	1													
	P	<0.001	<0.001	<0.001	<0.001														
Item 6	*r*	0.245	0.271	0.284	0.832	0.836	1												
	P	<0.001	<0.001	<0.001	<0.001	<0.001													
Item 7	*r*	0.136	0.124	0.149	0.182	0.182	0.189	1											
	P	0.007	0.014	0.003	<0.001	<0.001	<0.001												
Item 8	*r*	0.158	0.144	0.191	0.214	0.215	0.237	0.697	1										
	P	0.002	0.004	<0.001	0.012	<0.001	<0.001	<0.001											
Item 9	*r*	0.092	0.083	0.140	0.136	0.110	0.135	0.677	0.704	1									
	P	0.069	0.101	0.006	0.007	0.030	0.007	<0.001	<0.001										
Item 10	*r*	0.184	0.243	0.225	0.275	0.272	0.309	0.128	0.157	0.097	1								
	P	<0.001	<0.001	<0.001	<0.001	<0.001	<0.001	0.011	0.002	0.055									
Item 11	*r*	0.233	0.288	0.254	0.328	0.333	0.346	0.180	0.210	0.149	0.784	1							
	P	<0.001	<0.001	<0.001	<0.001	<0.001	<0.001	<0.001	<0.001	0.003	<0.001								
Item 12	*r*	0.200	0.236	0.210	0.303	0.302	0.341	0.159	0.192	0.148	0.786	0.873	1						
	P	<0.001	<0.001	<0.001	<0.001	<0.001	<0.001	0.002	<0.001	0.003	<0.001	<0.001							
Item 13	*r*	0.231	0.222	0.206	0.322	0.307	0.334	0200	0.295	0.228	0.235	0.291	0.272	1					
	P	<0.001	<0.001	<0.001	<0.001	<0.001	<0.001	<0.001	<0.001	<0.001	<0.001	<0.001	<0.001						
Item 14	*r*	0.205	0.207	0.205	0.304	0.266	0.291	0.214	0.268	0.238	0.226	0.257	0.245	0.838	1				
	P	<0.001	<0.001	<0.001	<0.001	<0.001	<0.001	<0.001	<0.001	<0.001	<0.001	<0.001	<0.001	<0.001					
Item 15	*r*	0.258	0.256	0.239	0.265	0.244	0.285	0165	0.215	0.195	0.204	0.261	0.243	0.820	0.814	1			
	P	<0.001	<0.001	<0.001	<0.001	<0.001	<0.001	0.001	<0.001	<0.001	<0.001	<0.001	<0.001	<0.001	<0.001				
Item 16	*r*	0.098	0.139	0.137	0.071	0.042	-0.012	0.119	0.078	0.071	0.249	0.206	0.198	0.111	0.114	0.077	1		
	P	0.052	0.006	0.007	0.161	0.403	0.814	0.018	0.126	0.162	<0.001	<0.001	<0.001	0.029	0.024	0.129			
Item 17	*r*	0.031	0.062	0.035	-0.018	-0.045	-0.103	0.068	0.031	0.060	0.193	0.162	0.138	0.080	0.098	0.050	0.873	1	
	P	0.540	0.222	0.488	0.716	0.378	0.041	0.181	0.541	0.233	<0.001	0.001	0.006	0.113	0.052	0.329	<0.001		
Item 18	*r*	0.062	0.081	0.068	0.048	-0.012	-0.053	0.136	0.077	0.101	0.226	0.194	0.180	0.157	0.173	0.115	0.844	0.852	1
	P	0.220	0.111	0.180	0.347	0.809	0.294	0.007	0.127	0.045	<0.001	<0.001	<0.001	0.002	<0.001	0.023	<0.001	<0.001	

*Note*. P, *p*-value; *r*, Pearson’s correlation coefficient.

### Exploratory factor analysis

The results of the EFA revealed that the SMS-II very well reflected the expected theoretical model with an overall good internal reliability. The internal reliability of the Arabic version of scale measured by McDonald’s omega, Cronbach’s alpha, and Gutmann λ6 values determined that it had good internal consistency (ω _SMS-II_ = 0.841, 95% CI = 0.818–0.864; α _SMS-II_ = 0.858, 95% IC = 0.835–0.878; λ6 _SMS-II_ = 0.952, 95% CI = 0.945–0.960). McDonald’s omega is a better indicator of internal reliability for the scale [52], as shown in Table 4. Internal consistency was excellent for all dimensions of the motivation (0.871 (IC 90%; 0.849–0.893) < ω < 0.948 (IC 90%; 0.939–0.957); 0.871 (IC 90%; .847–0.892) < α < 0.948 (IC 90%; 0.938–0.956); 0.819 (IC 90%; 0.764–0.860) < λ6 < 0.925 (IC 90%; 0.908–0.939)). Several statisticians [52–57] indicated the acceptable values for reliability coefficients higher at 0.60. As a result, most parameters had significantly high correlations with excellent values (see **Table 6**).

**Table 6:** Reliability coefficients of the sports motivation scale SMS-II.

		Cronbach’s α (CI 95%)	McDonald’s ω (CI 95%)	Guttman’s λ6 (CI 95%)
Sub-scales	IM	0.948 (0.938–0.956)	0.948 (0.939–0.957)	0.925 (0.908–0.939)
	Int.M	0.936 (0.925–0.947)	0.936 (0.925–0.947)	0.908 (0.886–0.925)
	Id.R	0.871 (0.847–0.892)	0.871 (0.849–0.893)	0.819 (0.764–0.860)
	Intro.R	0.924 (0.909–0.936)	0.924 (0.911–0.937)	0.892 (0.871–0.912)
	ER	0.933(0.921–0.944)	0.934 (0.922–0.945)	0.904 (0.884–0.920)
	AMO	0.947 (0.937–0.956)	0.947 (0.938–0.956)	0.923 (0.909–0.936)
SMS-II		0.858 (0.835–0.878)	0.841 (0.818–0.864)	0.952 (0.945–0.960)

*Note*. IM, intrinsic motivation; Int.M, integrated motivation; Id.R, identified regulation; Intro.R, introjected regulation; ER, external regulation; AMO, amotivation.

The results for all items supported the factor analysis (KMO = 0.819, Bartlett’s test of sphericity *p* < 0.001) and revealed six independent main factors with values above the threshold indicated by Cattell [58] and Kaiser [59], which explained 87.66% of the variance in the data. The clean value of the first major component of amotivation accounted for 30.73% of the total variance (eigenvalue = 5.53), while the second (intrinsic regulation) accounted for 15.45% (eigenvalue = 2.78), 12.17% (eigenvalue = 2.19), 11.02% (eigenvalue = 1.98), 9.91% (eigenvalue = 1.78), and 8.36% (eigenvalue = 1.50). Therefore, the first two independent main factors determined 46.18% of the total variance. We considered all except the dimensions that explained more than 1 [60].

For EFA, factor saturations of the six-factor model items were between 0.872 and 0.952 was depicted in **Table 7**.

**Table 7:** Standardized solutions for factor loadings for the sports motivation scale SMS-II.

SMS-II items	Components					
	1	2	3	4	5	6
1. لأنه يسعدني معرفة المزيد عن رياضتي		0.931				
Because it makes me happy to know more about my sport.						
2. لأنه من المثير للاهتمام معرفة كيف يمكنني التحسين		0.935				
Because it is so interesting to know how I can improve.						
3. لأنني أجد أنه من الممتع اكتشاف استراتيجيات جديدة للأداء		0.922				
Because I find it pleasurable to discover new performance strategies.						
4. لأن ممارسة الرياضة تعكس جوهر من أنا			0.908			
Because practicing sports reflects the essence of whom I am.						
5. لأنني من خلال الرياضة، أعيش وفقاً لمبادئي العميقة			0.909			
Because through sport, I am living in accordance with my deep principles.						
6. لأن المشاركة في الرياضة جزء لا يتجزأ من حياتي			0.896			
Because participating in sport is an integral part of my life.						
7. لأنني اخترت هذه الرياضة كوسيلة لتطوير نفسي						0.875
Because I have chosen this sport as a way to develop myself.						
8. لأنها من أفضل الطرق التي اخترتها لتطوير جوانب أخرى من نفسي						0.872
Because it is one of the best ways, I have chosen to develop other aspects of myself.						
9. لأنني وجدت أنها طريقة جيدة لتطوير جوانب من نفسي التي أقدرها						0.884
Because I found it is a good way to develop aspects of myself that I value.						
10. لأنني سأشعر بالضيق تجاه نفسي إذا لم آخذ الوقت الكافي للقيام بذلك					0.890	
Because I would feel bad about myself if I didn’t take enough time to do it.						
11. لأنني أشعر بتحسن تجاه نفسي عندما أفعل ذلك					0.893	
Because I feel better about myself when I do it.						
12. لأنني لن أشعر بأي قيمة إذا لم أفعل ذلك					0.908	
Because I wouldn’t feel worthwhile if I didn’t do it.						
13. لأن الناس من حولي يكافئونني عندما أفعل ذلك				0.903		
Because people around me reward me when I do that.						
14. لأنني أعتقد أن الآخرين سوف يرفضونني إذا لم أفعل ذلك				0.909		
Because I think others would reject me if I did not.						
15. لأن الأشخاص الذين أهتم بهم سينزعجون مني إذا لم أفعل ذلك				0.911		
Because the people I care about would be upset with me if I didn’t.						
16. حتى يمدحني الآخرون لما أقوم به			0.943			
So that others praise me for what I do.						
17. لم يعد واضحًا بالنسبة إلي، لا أعتقد حقا أن مكاني هو الرياضة			0.952			
It is not clear to me anymore; I don’t really think my place is in sport.						
18. كان لدي أسباب وجيهة لممارسة الرياضة، لكنني الآن أسأل نفسي إذا كان ينبغي علي الاستمرار			0.934			
I used to have good reasons for doing sports, but now I am asking myself if I should continue.						

### Confirmatory factor analysis

The six-factor model statistics are: χ^2^ = 144.591, 120 degrees of freedom at *p* > 0.063; CFI = 0.99; NFI = 0.97; TLI (NNFI) = 0.99; PNFI = 0.76; PCFI = 0.78; GFI = 0.96; AGFI = 0.94; SRMR = 0.02 and RMSEA = 0.02 (90%CI = 0.01–0.03).

For CFA, chi-square and χ^2^ normalized (χ^2^/df) statistics, the values obtained were good for the model as recommended by Wheaton, Muthen [61], Hermann, Joreskog [62], and Tabachnick and Fidell [63]. However, these authors value a set of indices (AGFI, GFI, CFI, TLI (NNFI), NFI, PNFI, PCFI, RMSEA, and SRMR) and suggest that the critical values for AGFI, GFI [63], NFI, CFI, and TLI must be greater than 0.95 [45,64–66]. For the RMSEA and SRMR, the index must be less than 0.05 and 0.08 for an acceptable fit, respectively, according to some scholars [44,67–69]. Generally, the results were satisfactory with the AGFI, GFI indices above 0.91 and the CFI, NFI and TLI (NNFI) values above 0.96, which implied that this model seemed to fit well. PNFI and PCFI exceeded 0.76. Therefore, the calculated values indicated a good fit with values. The SRMR and RMSEA were all below 0.02 showing a perfect fit. Therefore, CFA showed better adjustments for the Arabic six-factor SMS-II model.

In conclusion, the 18-item model revealed for all the indices tested an excellent fit to the theoretical model, justifying the six-dimensional factorial structure for a sample of Tunisian athletes (**Fig 2**).

**Fig 2:** Standardized results of the confirmatory factor analysis (CFA) of the Arabic version of SMS-II.

### Sensitivity analysis

From the results of the ANOVA, the sensitivity analysis indicates that team sports athletes between the ages of 13 and 18 years had more motivation to athletes in individual sports. While, individual sports athletes between the ages of 19 and 30 years used intrinsic motivation and introjected regulation more than athletes in team sports. There was also the effect of some variables (i.e., age, sport type) on introjected regulation and gender on external regulation. There was also another effect of sport type on identified regulation. On the other hand, in terms of effects of interaction, no significant influence could be identified (reported in **Table 8**).

**Table 8:** Impact of age, sex, sport type (i.e., team sports versus individual), and their inter-action effects on the dimensions of the motivation scale in sport (SMS‐II).

Variables	F					
	IM	Int.M	Id.R	Intro.R	ER	AMO
Age	0.105	6.537**	0.034	7.039**	0.556	0.071
Gender	1.349	0.331	0.205	0.221	4.954*	2.297
Sport	0.841	1.101	4.854*	8.446**	1.011	1.144
Age X Gender	1.782	3.550	0.032	2.406	0.265	1.270
Age X Sport	0.917	0.024	0.536	0.255	0.343	0.191
Gender X Sport	0.176	3.461	0.012	0.005	3.488	0.127
Age X Gender X Sport	2.675	1.084	0.613	0.330	0.379	1.389

*Note*. IM, intrinsic motivation; Int.M, integrated motivation; Id.R, identified regulation; Intro.R, introjected regula-tion; ER, external regulation; AMO, amotivation

* (*p* < 0.05)

** (*p* < 0.01).

## Discussion

In summary, the results of this study indicated that the Arabic version of the SMS-II is a reliable and valid tool for measuring the level of motivation in sport for athletes from both sexes and different types of sport (individual or team). Overall, we found very good psychometric properties for this adapted instrument. Moreover, the results collected by the EFA showed that this SMS-II scale well suggested the desired theoretical model, with good internal consistency for all the adopted dimensions. The 18 items of the SMS-II justified high reliability (McDonald’s omega = 0.841, Cronbach’s α = 0.858, Gutmann’s λ6 = 0.952) and excellent temporal stability (ICC = 0.960; *r* = 0.93, *p* < 0.001). Likewise, the CFA fit indices were good (CFI = 0.99; NFI = 0.97; CFI = NNFI (TLI) = IFI = 0.99; GFI = 0.96; AGFI = 0.94, and SRMR = RMSEA = 0.02).

The Sports Motivation Scale (SMS-28) remains less reliable in the sports context despite all the validations of this instrument in several languages: Greek [70], Spanish [71], German [72], Italian [73], Arabic [74], Polish [75] and Czech [76]. However, Pelletier, Vallerand [21] in SMS-6 as well as Lonsdale, Hodge [22] in the QSRB recommended changes to the scale. Researchers addressed the composition of the instrument and the nominal validity of sub-scales. They found that some components were no longer consistent with TDS. Regarding its development, the integrated regulation was included in the revised SMS-II version. These authors have shown that different forms of intrinsic motivation make the scale less reliable. Therefore, it is necessary to add other sub-scales valuing intrinsic motivation for this revised version to strengthen its structure and develop profitability. The scale was designed to assess athletes’ level of motivation for sport regarding SDT [20].

Moreover, the findings suggest of the EFA suggested that this measurement instrument well represented the desired theoretical model with good internal consistency for each dimension obtained. In our study, collected results indicated that the Arabic version of the SMS-II scale is a reliable and valid instrument for measuring athletes’ motivation in different disciplines. Our results reveal that the SMS-II scale [20] has good temporal stability and internal consistency. These studies have been confirmed by other researchers [16,23–27].

Concerning internal consistency, the reliability coefficients (i.e., McDonald’s ω, Cronbach’s α, and Gutmann’s λ6) measure the internal consistency of several items corresponding to a domain, i.e. the strength of the inter-correlations between items of the same domain (the homogeneity of the items). The more items are associated with each other, the closer the alpha coefficient is near 1.

Temporal stability of the questionnaire comprises controlling the resemblance of the same person’s answers to the questionnaire, at different times, but in the same experimental state. The statistical correlation between scores received during various times of answering the questionnaire is examined [65,77]. The correlation between two elements is perfect if it is 1. Therefore, the inter-scale correlations of our work were good. Intra-class Correlation Coefficients (ICC) with 95% confidence intervals were identified to justify the absolute agreement between the two moments. The SMS-II was constant over time over a one-month period. The absolute agreement between scores at both times with ICC with 95% confidence intervals and a 2-way random effects model was determined by a mean score (k = 2) of SMS-II [78].

The results of the CFA confirmed a good fit to the theoretical model, justifying the satisfactory six-dimensional factor structure in a sample of Tunisian athletes.

Finally, the results of our study confirm that there is a Tunisian version of the SMS-II with good psychometric properties, respecting the six-factor structure proposed by Pelletier, Rocchi [20] to measure the level of motivation in sport in Tunisia, which represents a step forward for sport psychology in the creation of a measurement tool for all sport type and for both sexes.

Athletes after age 30 have variety motivations, and it appears that motivations for engagement in sport may vary throughout the lifespan [79]. The athlete’s motivations affect performance in sport [80]. In the Arab world, studies that focus on motivation in the context of sport remain rare. It is advisable to use this instrument to learn about the importance of the motivational levels of athletes of both sexes and various ages.

However, our research had some limitations. It was necessary to conduct further validations with other instruments (basic needs satisfaction scale) since the athletes also passed through a continuum of adaptation in the activity (i.e., beginner, expert, or professional) which acted on their response. Arab validation could be influenced by Arab world culture, so it is necessary to share this validation with other countries to accommodate cultural changes and examine the general extensibility of athlete outcomes.

## Conclusion

Our work aimed to adapt the factorial structure, internal reliability, validity, and sensitivity of the SMS-II. The analysis revealed adequate temporal stability (test-retest), excellent internal reliability, perfect correlation values, good EFA factor structure, and excellent CFA adjustment indices. In terms of sensitivity, the analysis identified the impact of some variables (i.e., age, gender, and sport type) on some factor scores of motivations in sport. Therefore, our results indicated that the scale has good psychometric properties to measure the level of motivation for sport (whether collective or individual) in the Arab world.

## Supporting information

S1 Data Data of the 780 athletes. (XLSX)

S2 Data Data SMS-II-EFA (N = 390). (XLSX)

S3 Data Data SMS-II-CFA (N = 390). (XLSX)

S1 File Arabic version and original version of SMS-II. (DOCX)
